RETRACTED

# High-Intensity Injury Recognition Pattern of Sports Athletes Based on the Deep Neural Network

**DOI:** 10.1155/2022/2794225

**Published:** 2022-08-10

**Authors:** Nan Chen, Yang Zhang

**Affiliations:** ^1^Anyang Institute of Technology, Anyang, Henan 455000, China; ^2^Department of Physical Education, Shandong Jianzhu University, Jinan Shandong 250101, China

## Abstract

In order to solve the problem of low efficiency and accuracy of injury image recognition for sports athletes in high-intensity injury treatment, this paper proposes an injury recognition mode based on the deep neural network. In this paper, the image of sports injury is converted to gray level, and the contour of the injury part in the image is extracted according to the combination of adaptive thresholding and mathematical morphology. In this model, the seed points are selected, the active contour is used to approximate the initial contour, and the curve fitting method is used to fit the obtained discrete points to obtain the final damaged contour. The digital matrix is constructed by using the extracted number of pixels at the damaged position and relevant information. The images are arranged into feature vectors with a length of 64 according to the mode of column concatenation. The overall mean vector of the image is calculated. The calculation results, training samples, and image samples to be recognized are substituted into the Euclidean distance to obtain the preliminary recognition results of the damaged position of the image of sports injury. Then, the image segmentation is realized by clustering. The clustering segmentation results are used to color describe the pixel categories of the original image, calculate the relative damage proportion area in the sports injury image, and identify the damage parts of the high-intensity sports injury image. The experimental results show that the recognition rate of the neural network is 80%-100%, and the recognition time of this method is 0-0.6/s. The above method can improve the accuracy of the recognition of the damaged part of the sports injury image and shorten the recognition time and has certain feasibility in determining the sports injury part.

## 1. Introduction

After high-intensity training, athletes will inevitably suffer a certain degree of body damage, and athletes will continue to repeat a certain action, which will also cause wear and tear of body joints or skin [1]. For example, a competitive diver can be kept for a short period of time. The diver jumps from a high table, causing heavy movement in the air and eventually falling into the water. Throughout the procedure, all parts of the diver's body are injured [2].

RETRACTED

Not only the diving athletes but also the winter ice and snow athletes are seriously injured. Athletes often have injuries in relevant parts in winter sports, such as waist and back sports injuries, knee and ankle injuries, and large and small leg muscle injuries. Winter sports have higher technical requirements for athletes. In the day-to-day single training, athletes are easy to cause excessive load on the sports parts, resulting in lumbar muscle strain, ankle injury, and knee injury (Figure 1). The analysis of the survey results shows that the muscle and ligament injuries of winter sports athletes during exercise are consistent with the sports injuries of the patients included in this study. In this study, the patients' waist, back, knee, and ankle injuries had the highest probability, followed by shoulder, wrist, and leg injuries. In the process of daily training or competition, athletes' bodies are often kept at low temperature, and their muscles are easy to stiffen rapidly. When they do strenuous exercises to contract their muscles, they may cause muscle strain due to excessive strength and may also cause damage to the auxiliary tissues around the muscles. Because the distribution of blood vessels and muscles in the knee and ankle joints is less, they are prone to fatigue and slow recovery, so athletes are prone to sports injury in these two parts. The injury rate of athletes in daily training was 55.2%, and that in event competition was 36.8%. In addition, different sports and different injuries of athletes also have correlation. The sports injuries of ice athletes mainly occur in the waist, back, and limb joints. Therefore, in the process of sports, athletes' psychological pressure is greater, and the speed and impact are more intense than ordinary sports. Further analysis found that the main injury type of athletes was joint sprain, followed by muscle strain, which was consistent with other research results at home and abroad. The probability of sprain in winter sports is the highest, followed by abrasions, falls, and bumps. The characteristics of winter sports are related to the types of injury. Ice athletes have high technical requirements, high speed, and great difficulty and are prone to fall, impact, and fall or crash. Snow athletes are prone to crash or fall when they encounter road obstacles in training or competition. In addition, due to the low temperature in winter, if winter athletes do not keep warm or for other reasons, the blood flow in the body is not smooth, and they are prone to frostbite on the face, hands, and feet.

Many athletic events during athletic training involve high performance, and due to the repetition of training, some injuries are often eroded [3]. Injury must be treated. Determining the location of a wound in a wound image can help improve the outcome of treatment [4].

RETRACTED

In conclusion, it is necessary to identify the damage of the image of the athlete with the injury, to repair the injury, and to suggest ways to treat the injury. Research and analysis of wounds have been the focus of research in many areas [5]. Therefore, this paper provides a model for identifying injuries based on the deep neural network.

## 2. Literature Review

Based on the success of big data analysis, the deep neural network and its training algorithms have become well known in education and industry. Compared with traditional processes, in-depth studies are based on data and can extract objects (knowledge) from data. They have the advantage of analyzing large files of nonexistent, unambiguous, modified patterns, and names. The deep neural network currently used in big data analysis is usually a neural communication network, which is the advantage of creating static data and suitable for distributed according to application options. However, due to its limited structure, its ability to decompose temporary data is limited. An infinitely deep neural network is a type of frequency neural network with feedback connection. Basically, it is a dynamic system. Changes in the state of the network over time are important to this network. This is combined with “time loss,” which is necessary for extracting data over time series products and estimating large data. The conceptual model of this network expands over time. With the operation of time, this network can be “infinite depth,” so it is called an infinite depth neural network. In recent years, the infinite depth neural network computing method based on the restorative network structure has attracted more and more attention and has quickly become a research hotspot. It can be seen that the infinite depth neural network has great potential in processing time series data, and its powerful computing power in big data analysis and prediction tasks is increasingly apparent. As “big data analysis combined with intelligent computing” has become a research hotspot in the big data era, more new theories and methods in the field of infinite depth neural network computing will be proposed, and its application effect will be constantly refreshed, promoting the development and innovation of big data analysis technology.

Di and others have devised a method of examining wounds based on the characteristics of isolation and ultrasound. The results of the removal of the negative characteristics are achieved by analyzing the separation, and the completion process can be combined with LIBSVM to determine the damage [6]. Experimental results show that this method is effective, but the overall validity is low. Zhang and others devised a treatment based on the spectral improvement group [7]. Parida and others use multidimensional gray entropy based on similar characteristics to obtain a sample point spectrogram based on the analysis of the characteristics of the adjacent space and achieve the reduction in the weight of the spectrogram [8]. Beer and others argue that weight matching to the first lowest point in the statistical group is essential for the team to succeed. In order to reduce the loss of data to determine the damage, the process of calculating the value of self in spectral aggregation and obtaining better self-vectors was carried out [9]. Experimental results show that the level of data loss during error analysis is low, but the accuracy of the findings is not high. Hanteh and Rezaifar have proposed disaster management based on the wave coefficient Hu. HIFU is used to irradiate biological tissue, take B-ultrasound images before and after radiation, and take negative images [10]. A supporting vector technology is used to study and classify the structure of tissues by obtaining the results of wave coefficients and three percent values of the current subwave coefficients. Experimental results show that this method has some numerical accuracy, but the guarantee time is longer. Awareness of advanced trauma-based deep neural networks is recommended for athletes who use deep neural network devices to solve the problem of low accuracy and cognitive impairment.

RETRACTED

## 3. Method

### 3.1. Damage Image Processing

First, there must be a conversion on the sports map. For color images, the pixels can be represented by 3 bytes, and their corresponding bytes for lighting are made up of 3 elements, of which 3 elements are represented by R, G, and B. If the three components are the same, it is gray; otherwise, it is a color image. The formula for changing the grayscale value is as follows:

(1) $$\begin{array}{c} \text{Gray}\left(i,j\right)=0.299\cdot R\left(i,j\right)+0.587\cdot G\left(i,j\right)+0.114\cdot B\left(i,j\right). \end{array}$$

A 24-bit image does not change after conversion. An important role of replacing gray matter is to improve visual acuity [11].

### 3.2. Contour Extraction and Preliminary Recognition of Image Damage Location

In order to improve the accuracy of the defect detection, it is necessary to draw its contours. In this paper, mathematical morphology and adaptive thresholding methods will be used to create contours, and curves will be used to obtain broken contours [12]. The heavy injury contour design is a snake pattern that can receive the contour of the injured area. When the snake points in equilibrium, the energy is very small and the resulting contour coincides with the edge of the damaged area. Therefore, the contour strength must be reduced to a minimum in order to identify the damage. The two models for the contour movement expression are as follows:

(2) $$\begin{array}{c} E\left(C\right)=\left[\alpha E_{\text{in}}\left(C\right)+\beta E_{\text{ex}}\left(C\right)\right]\text{Gray}\left(i,j\right), \end{array}$$

where *α* and *β* represent weighted values and *E*_ex_(*C*) and *E*_in_(*C*) represent external energy and internal energy, respectively. Once the wound contour has been obtained, the site can be estimated using the K-L exchange method [13]. Once the contour has been removed, the number of pixels damaged and other important information can be obtained, so use this information to determine the digital matrix. In order to improve the accuracy of determining the location of the damage, it is necessary to place the images in 64 characteristic vectors that are arranged in a linear fashion. So there are *m* images, *X* = {*x*_1_, *x*_2_, ⋯, *x*_*m*_}, so formula (3) is for calculating the overall mean vector of images:

(3) $$\begin{array}{c} \mu =\frac{1}{m}\overset{m}{\underset{i=1}{\sum }}\;x_{i}\cdot E\left(C\right). \end{array}$$

Arrange the eigenvalues *A* in a decreasing manner. After the arrangement is completed, select the first *j* eigenvalues *λ*_*i*_ that are not zero, and then, extract their corresponding vector *v*_*i*_. Therefore, the covariance matrix eigenvector *μ*_*i*_ can be calculated according to formula (4). Select the first 60% of the eigenvalues, so that most of the damage images can be retained. In formula (4), *A* = [*x*_1_ − *μ*, *x*_2_ − *μ*, ⋯, *x*_*m*_ − *μ*].

(4) $$\begin{array}{c} u_{i}=A\frac{1}{\sqrt{\lambda_{i}}}X\cdot v_{i}\cdot \mu . \end{array}$$

Then, all the design drawings and training models that need to be decided are prepared in private space *U*, and the projection coefficient is calculated by

(5) $$\begin{array}{c} y_{i}=U^{T}\cdot u_{i}. \end{array}$$

Then, compare all the drawing models and training models to determine using equation (6). The model with the lowest spacing is the result of a preliminary analysis of the model [14].

(6) $$\begin{array}{c} d\left(x,y\right)={\left[\overset{n}{\underset{i=1}{\sum }}\;{\left(x_{i}-y_{i}\right)}^{2}\right]}^{1/2}. \end{array}$$

Here, *n* is the number of training patterns and *d* (*x*, *y*) is the Euclidean distance.

RETRACTED

### 3.3. Pixel Calculation of Damaged Image Based on the Neural Network

Through the above analysis, the damage location can be preliminarily identified, but the accurate location cannot be obtained. Therefore, the paper will further identify the damaged part by using the neural network, so as to obtain a more accurate damaged part and calculate the area of the damaged area [15].

Using the neural network in image damage recognition is to treat each solution as a fish, and then, all solutions form a solution set. There are two ways to find the final solution in the solution set: taking the cluster center as the solution and the cluster result as the solution. In order to improve the accuracy of the analysis, subgroups were used as a solution in this sentence [16, 17]. Therefore, the average vectors of each group are calculated for each fish, and the position of the fish can be used to represent one pixel in the image. Therefore, the target function of the fish can be indicated by the following model:

(7) $$\begin{array}{c} j_{g}=\overset{g}{\underset{i=1}{\sum }}\;{||V_{i}-x_{k}||}^{2}\cdot d\left(x,y\right), \end{array}$$

where *g* represents the number of cluster centers, *x*_*h*_ represents the cluster object, and *V*_*i*_ represents the pixel cluster centers. When *j*_*g*_ is the minimum value in the formula, it is set as the best clustering point, which is helpful to achieve the purpose of damage image segmentation [18].

After clustering, the gray pixel value of the image will reach the corresponding effect with the original pixel. After clustering results, the color rendering of pixels is realized, so different colors in the image will represent different representations. Thus, the RGB representation value of pixels can be calculated by accumulating the GRB flux of each type of pixel value and dividing it by the total number of pixels [19].

After the above analysis, the relative proportional area of the damage image can be expressed by

(8) $$\begin{array}{c} \text{ Are}{\text{a}}_{\text{ital}}=\left(\frac{W^{\prime }}{D^{\prime }}\right)\cdot 2.54\cdot \left(\frac{H^{\prime }}{D^{\prime }}\right)\cdot 2.54, \end{array}$$

where *D*′ represents the image resolution and *H*′ and *W*′ represent the number of pixels in different directions, with *H*′ representing the vertical direction and *W*′ representing the horizontal direction [20–22].

After clustering and segmentation of the original image, the area of the damaged area can be calculated through the correlation ratio, which is the ratio of the total number of damaged pixels *P* to the total number of image pixels *P*′, so formula (9) for the area of damaged pixels is as follows:

(9) $$\begin{array}{c} \text{ Are}{\text{a}}_{i}=\frac{P}{P^{\prime }}\cdot \text{Are}{\text{a}}_{\text{inal}}\cdot \min J_{g}. \end{array}$$

In the process of sports, athletes may have injuries at various positions of the human body, such as shoulder joint injuries, back injuries, and eye injuries. Through the above research based on the neural network, it can accurately identify the athletes' injury location and can improve the recognition efficiency. In order to further illustrate the accuracy and efficiency of this method, an experimental study will be carried out to verify its application effect.

RETRACTED

## 4. Results and Discussion

100 athletes were selected as subjects, and the relevant information of athletes is shown in Table 1.

The instrument is used to check the injury of each athlete in order to collect relevant data. Relevant data are obtained after the experiment, and then, the effect of damage image recognition based on the neural network is tested by using the recognition rate and recognition time.

1. Benefits of advanced research: to determine the effectiveness of self-assessment studied in this article, other assessments were selected as comparisons.  Figure 2 shows a comparison of the approvals of the different processes.  Figure 2(a) shows that the level of intelligence tends to change, first increases and then decreases, and its overall level decreases [23]. It can be explained that the research on the effectiveness of this method is flawed and it is not possible to determine the location of the loss, because the change in the rating level as can be seen in Figures 2(b) and 2(c) is also high. The level of acceptance of the assessment process studied in this sentence is better than that of the two methods, and the pattern of its changes is also similar. Recognition of sports images with serious injuries as neural connections allows athletes to first receive images of the injured area and then first identify the injury. The injury area is identified using K-L conversion analysis. Therefore, in order to verify authenticity, neural networks are used to divide the images and ultimately to obtain diagnostics with greater accuracy [24]. Therefore, the assessment process learned in this article is more feasible and robust than other methods
2. Recognition time-consuming analysis results: Figure 3 shows the time-consuming results of different recognition methods. It can be seen from the figure that when the number of images to be recognized is different, the recognition method based on the neural network takes the shortest time among the three methods. Therefore, it can be concluded that the method studied in this paper has faster recognition efficiency than the other two methods. Because the method has undergone image gray conversion before recognition, this step is conducive to improving the recognition efficiency [25]

The experiments shown in Figures 2 and 3 show that the plan has the advantages of both speed assurance and acceptance, and it can provide the basis strength and support for research in this area.

RETRACTED

## 5. Conclusion

This phrase provides a way to determine the severity of injuries in athletes based on deep neural networks. Athletes may be injured during sports. Determining their injury profile can help improve an athlete's performance in medical care. In this article, the damage of the image will be identified according to the neural network. Compared with the two methods of identification, the process in this document will help to improve the accuracy and authenticity of the analysis. Athletes can easily get injured during sports. In order to minimize injuries to athletes, we must adhere to strict operating standards to avoid serious injuries during training.

## Figures and Tables

**Figure 1:** Sports injury.

**Figure 2:** Recognition rate results of different methods.

**Figure 3:** Time-consuming results of different methods.

**Table 1:** Details of subjects.

Project	Remarks
Male/person	55
Female/person	45
Height range (cm)	162 ~ 183
Weight range (kg)	44 ~ 75
Training program	Weightlifting, sprinting, long-distance running, long jump, high jump, shot put, basketball
	Football, table tennis, javelin, etc.

## Data Availability

The data used to support the findings of this study are available from the corresponding author upon request.
